The article "Using Sociological Theories and Methods to Analyze the Solutions and Measures of Environmental Pollution Problems" was retracted in 2023. Reasons: signs of a paper mill; suspected computer-generated content; unreliable results or conclusions; concerns about the data.

# Using Sociological Theories and Methods to Analyze the Solutions and Measures of Environmental Pollution Problems

**DOI:** 10.1155/2022/9904222

**Published:** 2022-09-05

**Authors:** Suqin Chen

**Affiliations:** Party School of Lianyungang Municipal Committee of C. P. C., Lianyungang, Jiangsu 222006, China

## Abstract

In order to further improve the effectiveness of environmental pollution control and improve the quality of the atmospheric ecological environment, this article discusses regional environmental pollution control from the perspective of sociological theories and methods. Therefore, the article starts with the characteristics of environmental air pollution, combined with linear regression analysis and PSR model principal component analysis, focuses on the impact factors of environmental pollution, and concludes that the weights of pressure layer, state layer, and response layer for the impact of environmental state are 0.4824, 0.261, and 0.1207, respectively. On this basis, from the perspective of social, collaborative governance, and public management, this article focuses on the political measures of environmental pollution.

## 1. Introduction

At this stage, environmental pollution is an important topic of global research, and it is also a hot topic of common concern all over the world. The development of the world economy has brought about more and more serious air pollution problems (as shown in Figure 1). Environmental pollution-induced climate change and other hazards have seriously affected the health of the public and have gradually become an important obstacle to building a new face of modern social governance. Environmental pollution political work has also become the focus of the construction of a modern governance system of governments at all levels. Some local governments have carried out a series of air pollution control work in combination with national laws and regulations and the decisions of the central government and have taken a series of measures in combination with the actual situation of regional environmental pollution, and have achieved certain results. However, on the whole, the long-term social project of environmental pollution control needs to be adhered to for a long time in the aspect of pollution control. This study starts with the characteristics and impact factors of environmental pollution to explore long-term pollution control measures [1].

## 2. Literature Review

With the difficult situation of air pollution, the government has also increased the research on the countermeasures of air pollution control. The government should base itself on the law itself, improve the enforcement of the law, adopt a governance method independent of the government, adopt the establishment of professional institutions, and punish air pollution control, emission reduction, and violations. After recognizing that air pollution is dispersive in harmfulness, the government's legislation lags behind, and the means of implementation is single, it is difficult to effectively control air pollution only by legislative and other imperative policy tools. Howse et al. proposed reducing pollution sources in legal and administrative ways, encouraging emission reduction with market-oriented economic tools, and promoting the development of atmospheric governance and the environmental protection industry. Focus on promoting the use of environmental protection facilities and equipment and low consumption facilities and equipment, make full use of participatory policy tools and multichannel experts and citizens to participate, increase the number of governance participants, and announce and supervise the governance effect and other 10 air pollution governance issues. It can be seen that foreign scholars have studied the participation of air pollution control through policy tools since the middle of the twentieth century, especially the full use of three types of policy tools (command control, social participation, and economic incentive) to carry out pollution control research [2]. Liu et al. and others believed that “the cross regional joint governance of atmospheric environmental pollution should be implemented by adopting auxiliary green policies and measures during legislation,” reflecting the combined use of policy tools [3]. Luo et al., on the evaluation of government governance, believed that “the evaluation process of government governance policies is not limited to static discussion of existing government governance measures, but also combined with the improvement direction of government governance measures” [4]. Rodríguez et al. believed that in terms of air pollution control, while improving and integrating the implementation system of governance tools in the mode of government regulation in different regions, the particularity of air pollution control in different regions should be effectively enhanced, and the implementation quality of air governance in different regions should be improved based on an economic assessment means [5]. Sun and Wang, while focusing on the main policy tools of western countries to control fixed point source air pollution, focused on the analysis of China's policies to control fixed point source air pollution in the middle and lower reaches of the Yangtze River and their effects. On the basis of comparing the characteristics and applicable conditions of various types of policy tools, this article puts forward the adjustment and optimization methods of our government's policy choices in the future [6]. Anh et al. proposed that “we should make full use of the mandatory role of government public power to give play to the mixing of market economic means, stimulate the voluntary participation of different social organizations and the public, and solve the problem of the failure and deviation of government regulation in the air pollution control problem of this public policy problem” [7].

## 3. Analysis of Environmental Pollution Influencing Factors

### 3.1. Impact Analysis of Meteorological Factors on Air Quality Index

Taking a province as the research object, we plan to use meteorological factors such as average temperature (°C), relative humidity (%), precipitation (mm), and wind speed (m/s) to analyze the correlation of the monthly average AQI data of cities and prefectures in a province. In this section, the min-max normalization method suitable for small data scenarios is selected for processing. Data standardization refers to scaling factors of different orders of magnitude and units according to a certain proportion so that their change interval is transformed into [0, 1]. The standardized data value eliminates the problem of unit and value size and is conducive to the analysis of different indicators. Its standardized formula is as follows:

(1) $$\begin{array}{c} X^{\prime }=\frac{X-X_{\min}}{X_{\max}-X_{\min}}. \end{array}$$

In the above formula, *X*′ is a normalized vector with an interval of [0, 1], which belongs to a dimensionless pure digital form. *X* is the original data, and *X*_max_, *X*_min_ are the maximum and minimum values of the original data, respectively.

As shown in Figure 2, by analyzing the change trend between the monthly average of AQI and the monthly average of temperature after standardization in cities and prefectures of a province, it can be seen that during the period of high average temperature, the whole atmospheric environment is prone to strong convective weather, which will accelerate the dilution and transmission of pollutants by the atmosphere. Therefore, in the process of average temperature rising, the AQI value has a certain downward trend, and there is a strong negative correlation between the two.

As shown in Figure 3, by analyzing the change trend between the monthly average of AQI and the monthly average of precipitation after standardization in cities and prefectures of a province, it can be seen that in the season of high rainfall, pollutants in the atmosphere will be purified and diluted, and the greater the rainfall, the more significant the purification and dilution effect [8, 9]. Therefore, when the average precipitation rises, the corresponding AQI value has a certain downward trend, indicating that there is a strong negative correlation between the two.

As shown in Figure 4, the change trend between the monthly mean value of AQI and the monthly mean value of relative humidity after standardization in cities and prefectures of a province shows that in seasons with high relative humidity, pollutants are not easy to diffuse, and a large number of pollutants are attached to the air. Therefore, when the relative humidity rises, the corresponding AQI value also has a certain upward trend, indicating that there is a certain positive correlation between the two [10].

As shown in Figure 5, the change trend between the monthly mean value of AQI and the monthly mean value of the average wind speed after standardization in cities and prefectures of a province shows that a certain wind speed is conducive to the diffusion of pollutant concentration. When the average wind speed rises, the corresponding AQI value has a certain downward trend, indicating that there is a certain negative correlation between the two.

After comparing the change trend chart of AQI monthly mean with conventional meteorological factors (average temperature, precipitation, relative humidity, and average wind speed), it is found that the level of AQI monthly mean is related to the change of conventional meteorological factors to a certain extent. Based on the positioning of this logical relationship, a preliminary inference is made: AQI monthly mean is correlated with conventional meteorological factors. Using the bivariate analysis function in SPSS software, the correlation between AQI monthly mean and different conventional meteorological factors is tested respectively (see Table 1 for the results) so as to fit the optimal curve equation [11, 12].

Main calculation results and conclusions are as follows:

1. AQI monthly mean and average temperature show a significant negative correlation (double-tailed) on the 0.01 layer, and the correlation coefficient is −0.755.
2. AQI monthly mean is significantly negatively correlated with precipitation at 0.01 layer (double-tailed), and the correlation coefficient is −0.780.
3. AQI monthly mean is significantly positively correlated with relative humidity at 0.01 layer (double-tailed), and the correlation coefficient is 0.726.
4. The monthly average of AQI is significantly negatively correlated with the average wind speed on the 0.01 layer (double-tailed), and the correlation coefficient is −0.791.
5. The correlation coefficient between AQI monthly mean and conventional meteorological factors is arranged as follows: average wind speed > precipitation > average temperature > relative humidity.

### 3.2. Linear Regression Analysis

#### 3.2.1. Linear Regression Prediction

If the scatter plot of the data roughly shows a linear distribution, the equation of the prediction model is as follows:

(2) $$\begin{array}{c} Y=a_{0}+a_{1}X. \end{array}$$

#### 3.2.2. Curve Regression Prediction

If the scatter plot of the data shows a certain curve change law, the equation types of the prediction model are mainly as follows:

Logarithmic model:
  (3) $$\begin{array}{c} Y=a_{0}+a_{1}\text{In}X. \end{array}$$
Quadratic model:
  (4) $$\begin{array}{c} Y=a_{0}+a_{1}X+a_{2}X_{2}. \end{array}$$
Cubic model:
  (5) $$\begin{array}{c} Y=a_{0}+a_{1}X+a_{2}X_{2}+a_{3}X_{3}. \end{array}$$
Logistic model:
  (6) $$\begin{array}{c} Y=\frac{1}{\left(1/u+a_{0}a_{1}X\right)}. \end{array}$$
Index model:
  (7) $$\begin{array}{c} Y=a_{0}ea_{1}X. \end{array}$$

#### 3.2.3. Multiple Linear Regression Prediction

If there is more than one factor affecting the prediction index, the multiple regression equation should be used for data analysis. The equation of the prediction model is as follows:

(8) $$\begin{array}{c} Y=a_{0}+a_{1}X_{1}+a_{2}X_{2}+a_{3}X_{3}+...+a_{n}X_{n}. \end{array}$$

#### 3.2.4. Data Processing and Result Analysis

This section will evaluate the correlation between the overall air environmental quality (AQI) of a province and the standardized meteorological data and fit the corresponding linear regression equation using Pearson's correlation analysis, combined with the monthly routine meteorological factor data (average temperature, precipitation, relative humidity, and average wind speed) of cities and prefectures in a province from 2015 to 2017. Usually, the Pearson correlation coefficient between two continuous variables (*X*, *Y*) is defined as the quotient of the product of the covariance of the variable and the standard deviation. The specific form is as follows:

(9) $$\begin{array}{c} \rho_{xy}=\frac{\mathrm{cov}\left(x,y\right)}{\delta x\delta y}=\frac{E\left(x-\mu_{x}\right)\left(y-\mu_{y}\right)}{\delta x\delta y}, \end{array}$$

where *ρ*_*xy*_ represents the correlation coefficient of the variable and cov(*x*, *y*) represents the covariance of the variable. Among them, the sample correlation coefficient is defined as the covariance and standard deviation of the sample corresponding to the covariance and standard deviation of the population in the following form:

(10) $$\begin{array}{c} r=\frac{\sum_{i=1}^{n}\left(x_{i}-\bar{x}\right)\left(y_{i}-\bar{y}\right)}{\sqrt{\sum_{i=1}^{n}{\left(x_{i}-\bar{x}\right)}^{2}\sum_{i=1}^{n}{\left(y_{i}-\bar{y}\right)}^{2}}}, \end{array}$$

where *r*  is Pearson's correlation coefficient; *x*, *y* is the data variable; $\bar{x},\bar{y}$ is the mean value of variables *x*, *y*; *x*, *y* is the *i* th observation of variables *x*, *y*. When *r* > 0, the two continuous variables show positive correlation; when *r* < 0, the two continuous variables show a negative correlation. If the absolute value of the correlation coefficient is larger, it means that the correlation between variables is stronger. Since the value of the Pearson correlation coefficient is [−1, 1], when *r* = 1, it means that the variables are completely positive correlation; when *r* = −1, it means that the variables are completely negative correlation, and when *r* = 0, it means that there is no correlation between variables. There is a significant correlation between AQI monthly mean and average temperature, precipitation, relative humidity, and average wind speed. In order to explore the overall relationship between AQI value and conventional meteorological factors, we can analyze it by establishing a linear multiple regression equation, assuming that the multiple equation is as follows:

(11) $$\begin{array}{c} C=\partial_{0}+\partial_{1}T+\partial_{2}W+\partial_{3}P+\partial_{4}V. \end{array}$$

where *C* represents the AQI value, *∂*_0_ is the constant term, *∂*_1_, *∂*_2_, *∂*_3_, *∂*_4_ are the partial regression coefficient, and *T*, *W*, *P*, *V* represent the values of average temperature, precipitation, relative humidity, and average wind speed, respectively.  Table 2 shows the overall fitting of the established model 4, with a complex correlation coefficient (*R*) of 0.861, a goodness of fit *R*^2^ of 0.741, and a Durbin–Watson test statistic of 0.741, indicating that the residuals are independent [13–15].

As shown in Table 3, the observed value of the F statistic in the model is 13.594, and the probability sig (*P* value) is <0.01. Under the condition of a significance level of 0.05, it can be considered that C (AQI monthly mean) is linearly correlated with *t* (average temperature), *w* (precipitation), *P* (relative humidity), and *V* (average wind speed).

Table 4 shows various parameters in the model, such as partial regression coefficient (b), standard error (std.error), constant (constant), standardized partial regression coefficient (beta), t-statistic observation value of regression coefficient test, and corresponding probability *P* value (SIG). Based on this multiple model, the multiple linear regression equation between meteorological factors and AQI monthly mean can be obtained as follows:

(12) $$\begin{array}{c} C=103.406-8.537T-13.381W+7.614P-32.463V. \end{array}$$

Through the established linear regression equation (12), it can be seen that the monthly mean change of AQI in cities and prefectures of a province will be significantly affected by meteorological factors, and the influence degree of each meteorological factor on AQI is as follows: average wind speed > precipitation > average temperature > relative humidity.

### 3.3. PSR Model Construction Analysis

The index system under the PSR model is shown in Table 5.

In order to minimize the influence of subjective factors, this article will use principal component analysis to determine the weight. In this section, the principal component extraction will choose whether the cumulative variance contribution rate reaches 85% as the standard, which means to ensure that the amount of information contained in the principal component accounts for more than 85% of the original data, so that the amount of information lost is less than 15% [16].

In this article, the original data and the standardized data are replaced by P1–P10 and ZP1-ZP10, respectively, where ZP1-ZP3 is the pressure layer index data, ZP4-ZP8 is the state layer index data, and ZP9-ZP10 is the response layer index data. Before using SPSS software for correlation analysis, the KMO test and Bartlett's sphericity test were performed on the data, respectively. The test results are shown in Table 6.

Among them, the size of the KMO test value represents the strength of the correlation between the principal components, and its value range is between 0 and 1, while the size of the Bartley sphericity test value represents the strength of the independence between various variables. When the test results meet, the KMO test coefficient >0.5 and the significance probability (*P* value) of Bartley test value <0.05; it indicates that the correlation between the principal components is strong, and the selected dataset is suitable for principal component analysis, so the constructed PSR model can have complete structural validity for the next step of factor evaluation and analysis, in which the kmo test statistics are as follows:

(13) $$\begin{array}{c} \text{KMO}=\frac{\sum \sum r_{ij}^{2}}{\sum \sum r_{ij}^{2}+\sum \sum p_{ij}^{2}}. \end{array}$$

As shown in Table 7, taking the critical value 1 of the initial characteristic value as the standard, the initial values of the principal components required to be obtained are greater than 1. Through SPSS software calculation, a total of 3 principal components can be selected, which are identified as *Z*1, *Z*2, and *Z*3, respectively, and the cumulative variance contribution is 86.416%.

According to the numerical relationship between each index and the three principal components in the component score matrix (Table 8), the expression of the three principal components can be obtained:


(14) $$\begin{array}{c} Z_{1}=0.098*ZP_{1}+0.022*ZP_{2}+0.249*ZP_{3}-0.172*ZP_{4}-0.03*ZP_{5}\\ -0.025*ZP_{6}+0.124*ZP_{7}+0.142*ZP_{8}+0.279*ZP_{9}+0.303*ZP_{10},\\ Z_{2}=0.172*ZP_{1}+0.091*ZP_{2}-0.026*ZP_{3}+0.331*ZP_{4}+0.299*ZP_{5}\\ +0.298*ZP_{6}+0.01*ZP_{7}+0.056*ZP_{8}-0.059*ZP_{9}-0.155*ZP_{10},\\ Z_{3}=-0.037*ZP_{1}+0.51*ZP_{2}-0.011*ZP_{3}-0.013*ZP_{4}+0.001*ZP_{5}\\ -0.094*ZP_{6}+0.669*ZP_{7}+0.062*ZP_{8}-0.08*ZP_{9}-0.168*ZP_{10}. \end{array}$$

The corresponding index data of cities in a province are substituted into the expression to calculate the ranking of cities under each index benchmark and the ranking of 21 cities in a province in the pressure layer, state layer, response layer, and comprehensive index layer of the model. Among them, the higher the ranking of the pressure layer, the greater the environmental pressure faced by the representatives; the higher the ranking of the state layer, the worse the atmospheric environment quality; the higher the ranking of the response layer, the more sufficient the response measures taken on behalf of the government departments; the comprehensive index layer represents the comprehensive evaluation of the overall performance [17].

## 4. Environmental Pollution Remediation Measures from the Perspective of Social Collaborative Governance

### 4.1. Problems in Collaborative Treatment of Environmental Pollution

In order to understand the relevant situation of collaborative governance in the city, this article designs a questionnaire. Considering that different social subjects have different roles in the collaborative governance of air pollution, they have different perspectives on the collaborative governance of air pollution and different specific work contents. The questionnaire is distributed to government staff, business leaders, and the public. The distribution methods include paper and Internet, with 100 copies each, a total of 300 copies. The questionnaire was conducted anonymously, and the effective questionnaire rates were 92%, 87%, and 93%, respectively.

#### 4.1.1. Insufficient Horizontal Coordination between Government Departments

Although *L* City has issued the work responsibilities of various municipal departments in the field of environmental protection, the specific contents of the responsibilities are not detailed enough. More importantly, it has expanded and extended in the field of environmental protection from the perspective of the three fixed plans of the department. However, the actual work task is intertwined with many problems and aspects. Often, work involves multiple departments and requires the coordinated efforts of multiple departments. In this micropractical operation, the department's responsibilities are not clear. According to the questionnaire for government staff, 46% of the respondents believed that the clarity of responsibilities was “average,” 16% of the respondents believed that the clarity of responsibilities was “unclear,” and 38% of the respondents believed that the clarity of responsibilities was “clear” or “relatively clear” (Figure 6).

#### 4.1.2. The Synergy between the Government and the Public Is Poor

At present, the way of public participation in air pollution control in *L* City only stays at the letter and visit participation through the telephone network and other channels. *L* City has not yet established other diversified public participation systems, and the way of public participation only stays at the initial stage. The questionnaire to the public showed that 91% of the respondents believed that the government's dominance in the current air pollution control was “very high,” 18% of the respondents believed that the public's participation in the air pollution control was “poor,” and 74% of the respondents were “unclear” about the public's participation in the air pollution control, as shown in Figures 7 and 8.

The effectiveness of public participation is insufficient. Air pollution control is a systematic project, which requires the active cooperation of various subjects. In fact, although the public has a strong intention to participate and abhors pollution behaviors, they often fall into a situation where they are willing but unable [18]. Public participation is mostly in the form of individuals, generally acting alone and lack of organization. In practice, the participation ability can not effectively form a joint force, which leads to the lack of participation ability and affects participation efficiency. Moreover, public participation in air pollution control is at the end of the stage. Only when pollution occurs and produces obvious sensory discomfort, such as vision and smell, will it intervene, and the participation is too passive and lagging.

#### 4.1.3. Low Enthusiasm of Enterprises to Participate in Governance

The main source of air pollutants is the production and operation activities of enterprises. Enterprises are important producers of pollution, and enterprises must bear the main responsibility in air pollution control. On the one hand, there is an obvious lack of awareness of the social responsibility of enterprises to control pollution, and the lack of governance concept is relatively serious, although the state has legislated and issued policies to strengthen the main responsibility of enterprises and has taken a series of methods to increase the illegal cost of enterprises to effectively investigate the responsibility of enterprises for illegal emissions. However, the production of enterprises has the nature of giving priority to reducing costs and improving the return on capital, and the phenomenon of unwillingness to consciously perform or even avoid their own environmental and social responsibilities is still widespread. On the other hand, as a profit-making organization, enterprises pursue the maximization of economic interests and give priority to economic interests rather than social benefits. Participating in air pollution control will inevitably lead to an increase in enterprise operating costs and the reduction of profits, and even cause losses. At the same time, due to the publicity and nonexclusivity of the atmospheric environment, some enterprises have a strong “free rider” mentality. For the consideration of reducing the treatment cost and increasing profits, enterprises do not have a strong initiative and enthusiasm to carry out air pollution control.

### 4.2. Countermeasures to Improve the Effectiveness of Environmental Pollution and Social Collaborative Governance

#### 4.2.1. Clarify the Relevant Responsibilities of Various Departments within the Government

On the basis of establishing a highly authoritative air pollution control organization headed by the main responsible comrades of the Party committee and the government, we should strengthen field research, fully study the specific operability, scientificity, and feasibility of the control plan, further clarify the work content and scope of authority of relevant government departments in work, promote the meticulous and refined implementation of responsibilities, and try to avoid unclear rights and responsibilities the responsibility is unknown [19]. Establish awareness of the whole process, respond in time to different problems at different work levels, coordinate and communicate as soon as possible, enhance the predictability of work, change work methods, turn passivity into the initiative, and build a new and efficient comprehensive management system.

We will further promote the clarification of the rights and responsibilities of horizontal government departments and clearly determine the responsibilities and obligations of departments in air pollution control according to the situation that different departments are responsible for different air pollution sources. For example, the development and reform department is responsible for industrial access and resource consumption, the industry, and information technology department is responsible for the elimination of backward production capacity, the housing and construction department is responsible for the dust control of construction sites, the commerce department is responsible for the supervision of motor vehicles (ships) and oil products, the ecological environment department is responsible for the pollution control of industrial enterprises, and the urban management and law enforcement department is responsible for road cleaning and catering lampblack control, so as to form a list of departmental rights and responsibilities and reduce the buck passing between departments. At the moment of the reform of government institutions, combined with the current situation of unbalanced law enforcement power and uneven level of departments, it is necessary to break the barrier between department law enforcement, form a comprehensive and cross-department law enforcement agency, realize the integration of law enforcement, and make the flow of information more smooth. Make up for the defects of the current department law enforcement mode of fighting alone with the joint force of law enforcement, and expand the exchange and cooperation between departments to promote collaborative governance through the unification and innovation of the law enforcement supervision mode.

#### 4.2.2. Effectively Use Fault Tolerance and Error Correction Mechanism to Break the Dishwashing Effect

In air pollution control, we need to effectively use the fault-tolerant and error correction mechanism, break the negative impact of the dishwashing effect on government officials, remove the ideological burden that hinders government officials from innovating their working methods and shouldering the heavy burden, encourage officials to be brave in taking on responsibilities, bold in innovation, and actively act, and actively participate in the work of air pollution control based on their own job responsibilities. Establish both result orientation and process orientation. Officials who work steadily and conscientiously in accordance with the established work deployment and responsibility objectives will be exempted from accountability even if there are mistakes so as to form a good orientation and maintain the enthusiasm of officials. However, it is necessary to pay attention to the scope of application of the fault-tolerant mechanism so that it can really play a positive guiding role and avoid the use of the fault-tolerant mechanism to “loosen discipline,” “give mercy outside the law,” and take fault-tolerant as a “protective umbrella.” For those who do not act and act indiscriminately, they should be resolutely held accountable to form clear and correct guidance.

#### 4.2.3. Reform the Evaluation Methods and Increase the Proportion of Pollution Control

At present, although the government is not only a hero in the comprehensive assessment of economic and social development, economic development still occupies a leading position, and the proportion of environmental governance is still too small. Therefore, it is necessary to combine the new development concepts of innovation, coordination, green, openness, and sharing, optimize and adjust the content of the current performance appraisal, establish a more coordinated and specific performance appraisal method, and promote the change of the governance concept and thinking of officials with the optimization of the appraisal content. We should further improve the assessment method of air pollution control, increase the content of process assessment, and pay attention to the phased improvement of various assessment indicators in addition to legal assessment indicators. At the same time, we should implement the responsibility system of “the same responsibility of the party and the government, one post and two responsibilities” for environmental protection, and compact the responsibility of air pollution control to party committees and governments at all levels and departments, so as to force them to perform their duties. We should build a performance appraisal and accountability model focusing on major government officials and pay attention to the construction of a responsibility system, such as implementing the departure audit system for natural resource assets of leading cadres, establishing a lifelong accountability system for ecological environment damage, and exploring the establishment of a government natural resource balance sheet system. We should truly combine the effectiveness of air pollution control with the selection and appointment of leading cadres to achieve “the best, the mediocre, and the worst” and improve the effectiveness of local government environmental governance.

#### 4.2.4. Strengthen the Participation of Other Subjects

First, both government regulatory information and unit emission information are made public.
The supervision of the society, media, and the public is the best way of supervision, and it is also an effective way to encourage the government and pollutant discharge units to perform their duties in strict accordance with the relevant requirements. The government's relevant information disclosure is also a key measure to protect the public's right to know. The government needs to increase the detailed information disclosure on air pollution control to make the environmental situation as comprehensive as possible known to the public. Continue to unswervingly promote the disclosure of government information and try to achieve the goal of “openness is the norm and nonopenness is the exception” in accordance with the requirements of the State Council, so that the government can work in the sun, and the whole process of work deployment, implementation, operation, and evaluation is transparent, and consciously accept supervision in the vision of society, the media, and the public. Give play to the guiding and publicity role of government information disclosure, build new and effective ways of communication and connection, and reduce the cost of public access to the atmospheric environment in all aspects. Constantly enrich the public information content; especially the information related to examination and approval, planning, and other sensitive aspects must be made public as much as possible. Continue to expand the communication channels of information disclosure, not only in the regular communication channels but also in the mobile terminals with a high frequency of public use, such as Weibo and apps, so as to improve the acceptance of information disclosure and fully reflect the effectiveness of government information disclosure. At the same time, due to the strong professionalism of air pollution control, the government also needs to establish a platform to popularize science to the public and improve the professionalism of the public. On the other hand, pollutant discharge units also need to strengthen the awareness of information disclosure, avoid refusing to disclose information on the grounds of trade secrets, and must disclose accurate pollutant discharge information to the public, subject to the supervision of relevant government departments and the supervision of all sectors of society [20].
Second, use policies, finance, and other means to encourage enterprises to control pollution.
    Firstly, strictly implement the principle of “whoever pollutes, who governs,” and bring enterprises into the framework of the ecological compensation system. Clarify the provisions of the corresponding polluters, stakeholders, and other parties, build a mechanism that causes cost pressure on enterprise emissions, control the total emission of air pollutants, and reward enterprises that discharge air pollutants with high standards, and the polluters bear their own responsibilities and compensate the stakeholders.
    Secondly, implement emissions trading. In this regard, we can learn from some foreign advanced experience and use market means to let enterprises consciously take measures to limit the emission of air pollutants. It can also reduce the emission cost of enterprises and reduce the possible adverse impact of air pollution control on the economy. At the same time, the implementation of an emission trading system can also promote the unification of pollutant emission standards of enterprises and contribute to the effective promotion of air pollution prevention and control related work.

## 5. Conclusion

This study first analyzes the changes of the city as a whole, regional distribution, and different time nodes of the pollution indicators of cities in a province from two different dimensions of time and space. Secondly, the correlation analysis, regression analysis, and superposition analysis of the overall pollution situation in a province are carried out by collecting the ground meteorological factor data (average temperature, precipitation, relative humidity, and average wind speed) and digital elevation data (DEM) in the corresponding period. Finally, based on the preliminary understanding and mastery of the spatial and temporal characteristics of air pollution in cities in a province, in order to further clarify the causes and mechanisms of how human activities cause air pollution, the air pollution evaluation system of cities in a province is constructed by establishing a PSR (pressure state response) model. The weight of the pressure layer, state layer, and response layer on the impact of the environmental state is 0.4824, 0.261, and 0.1207, respectively. Secondly, using the theory of collaborative governance, this article analyzes the problems existing in the two aspects of government internal collaboration and government social public collaboration in the air pollution governance of *L* City and finally puts forward countermeasures and suggestions. That is to clarify the internal responsibilities of the government, deepen the supervision and promote the implementation of departmental responsibilities, effectively carry out fault tolerance and correction, reform the assessment and evaluation, promote the research and production of pollution control, make the government regulatory information and the unit emission information both public, use policy and financial means to stimulate enterprises, mobilize public participation enthusiasm through multiple channels, and work together internally and externally, providing a certain reference for *L* City's air pollution control.

## Figures and Tables

**Figure 1:** Environmental pollution.

**Figure 2:** Change trend of monthly average AQI and temperature range after standardization in a province.

**Figure 3:** Variation trend of monthly average AQI and precipitation interval after standardization in a province.

**Figure 4:** Variation trend of monthly average AQI and humidity range after standardization in a province.

**Figure 5:** Variation trend of monthly average AQI and wind speed range after standardization in a province.

**Figure 6:** Horizontal collaboration survey results between government departments.

**Figure 7:** The leading degree of the government in the current collaborative control of air pollution.

**Figure 8:** Public participation in the process of air pollution control.

**Table 1:** Factor correlation coefficient.

Variable	1	2	3	4	5
AQI	1				
Average temperature	−0.755^*∗∗*^	1			
Precipitation	−0.780^*∗*^	0.859^*∗∗*^	1		
Relative humidity	0.726^*∗∗*^	−0.842^*∗∗*^	−0.873^*∗∗*^	1	
Average wind speed	−0.791^*∗∗*^	0.757^*∗∗*^	0.608^*∗∗*^	−0.728^*∗∗*^	1

Note: ^*∗*^*P* < 0.05, ^*∗∗*^*P* < 0.01, ^*∗∗∗*^*P* < 0.001.

**Table 2:** Model factors.

Model	*R*	*R* ^2^	Adjusted *R*^2^	Error of standard estimation	Durbin–Watson
4	0.861	0.741	0.687	9.634	0.741

**Table 3:** Residual analysis table.

Model		Sum of squares	Degrees of freedom (d*f*)	*F*	Significance
4	Regression	5047.162	4	13.594	<0.01
	Residual	1763.528	19		
	Total	6810.690	23		

**Table 4:** Regression coefficient table.

Model	Coefficient of nonstandardization		Standardization coefficient	*t*	Significance
	*B*	Standard error	Beta		
Constant	103.406	16.200	6.383	<0.01	
Temperature	−8.537	17.861	−0.137	−0.478	<0.01
Precipitation	−13.381	14.158	−0.258	−0.945	<0.01
Relative humidity	7.614	14.614	0.139	0.521	<0.01
Average wind speed	−32463	14.996	−0.411	−2.165	<0.01

**Table 5:** Index system based on PSR model.

Target layer	Project level	Index layer
Atmospheric pollution scenario simulation	Pressure layer	Population density (person/km^2^)
		Per capita GDP (yuan)
		Proportion of secondary industry in total GDP (%)
		AQI index
	State layer	Average annual mass concentration of PM_25_ (*μ*g/m^3^)
		Average annual mass concentration of PM_10_ (*μ*g/m^3^)
Atmospheric pollution scenario simulation	State layer	Annual average mass concentration of SO_2_ (*μ*g/m^3^)
		Annual average mass concentration of NO_2_ (*μ*g/m^3^)
	Response layer	Vehicle ownership (10000)
		Park green area (square kilometers)

**Table 6:** KMO and Bartlett's sphericity test.

Kaiser–Meyer–Olkin	Measurement and sampling suitability	0.618
Bartlett's sphericity test	Approximate chi-square d*f*	237.883
		45
	Significance (sig.)	<0.01

**Table 7:** Total variance explained.

Initial characteristic value				Extract sum of squares load			Rotation sum of squares loading		
Component	Total	% of variance	Cumulative%	Total	% of variance	Cumulative%	Total	% of variance	Cumulative%
1	4.824	48.242	48.242	4.824	48.242	48.242	3.978	39.783	39.783
2	2.61	26.1	74.342	2.61	26.1	74.342	3.205	32.051	71.835
3	1.207	12.073	86.416	1.207	12.073	86.416	1458	14.581	86.416
4	0.575	5.745	92.161						
5	0.312	3.117	95.278						
6	0.214	2.143	97.421						
7	0.149	1.493	98.913						
8	0.074	0.736	99.649						
9	0.034	0.337	99.986						
10	0.001	0.014	100						

**Table 8:** Component score matrix.

Indicator type	Component		
	1	2	3
*Z*_score_ (population density)	0.098	0.172	−0.037
*Z*_score_ (per capita GDP)	0.022	0.091	0.510
*Z*_score_ (proportion of secondary industry)	0.249	−0.026	−0.011
*Z*_score_ (AQI)	−0.172	0.331	−0.013
*Z*_score_ (PM_25_)	−0.030	0.299	0.001
*Z*_score_ (PM_10_)	−0.025	0.298	0.094
*Z*_score_ (SO_2_)	−0.124	−0.01	0.669
*Z*_score_ (NO_2_)	0.142	0.056	0.062
*Z*_score_ (vehicle ownership)	0.274	−0.059	−0.080
*Z*_score_ (park green area)	0.303	−0.155	−0.168

## Data Availability

The labeled dataset used to support the findings of this study is available from the corresponding author upon request.
